The article "Application of multimedia technology to innovative vocational education on learning satisfaction in China" was retracted in 2024. Reasons: concerns about the data; concerns about the results or conclusions; concerns about the authorship; concerns about the welfare of human subjects.

# Application of multimedia technology to innovative vocational education on learning satisfaction in China

**DOI:** 10.1371/journal.pone.0298861

**Published:** 2024-02-28

**Authors:** Shengnan Wu

**Affiliations:** Academic Affairs Office, Beijing Institute of Economics and Management, Beijing, China; Tallinn University: Tallinna Ulikool, ESTONIA

## Abstract

Multimedia technology holds paramount importance in driving innovation within vocational education, significantly influencing learning satisfaction. Its integration facilitates dynamic and interactive learning environments, catering to diverse learning styles and preferences. Moreover, multimedia technology enables educators to simulate real-world scenarios, providing practical and hands-on training opportunities. This aspect is particularly valuable in vocational education, where practical skills and application are required. The paper investigates the impact of multimedia technology in enhancing learning satisfaction within innovative vocational education. It delves into the utilization of multimedia tools and their correlation with learner satisfaction, exploring how these technologies augment engagement and comprehension in vocational training. The primary data from 515 students of vocational colleges of China has been collected and regression analysis is applied for empirical analysis. The findings of the study highlight that multimedia technology has positive relationship with innovative vocational education and learning outcome. The findings contribute valuable insights for policymakers regarding significant role multimedia plays in fostering enhanced learning experiences and overall satisfaction among vocational learners.

## 1. Introduction

The relationship between technology and vocational education is dynamic and impactful, shaping the way vocational skills are taught, acquired, and applied in various industries [1]. Technology integration in vocational education aligns teaching with industry standards. It allows students to familiarize themselves with the tools and equipment used in their specific fields, ensuring they are job-ready upon graduation [2]. Technology enriches the learning experience by providing interactive simulations, virtual labs, and online resources [3]. Online platforms and digital resources provide access to specialized knowledge and expertise from around the world. This widens the scope of learning beyond geographical limitations, allowing students to access the latest information and advancements in their fields [4]. As technology evolves, vocational education adapts to include emerging skills demanded by future job markets [5]. Courses on robotics, AI, cybersecurity, and other tech-related subjects are integrated into vocational curricula to prepare students for evolving industries [6]. Technology is an integral part of vocational education, enhancing skill development, customization of learning experiences, access to global knowledge, industry alignment, flexibility, and innovation in teaching methods [7]. This relationship continues to evolve, ensuring that vocational education remains relevant and adaptive to the changing demands of the workforce [8].

There are numerous shortcomings and challenges persist in the integration of multimedia technology in most vocational colleges. These issues are reflected in various aspects. Firstly, the potential of multimedia, as a relatively modern teaching method, remains underutilized and impeding its full efficacy. Secondly, many vocational institutions continue to employ traditional educational approaches, resulting in significant discrepancies and challenges in integration of multimedia technology and hindering its optimal application. Additionally, innovations through vocational education and satisfaction of students rely heavily on knowledge-based metrics but there is lack of a comprehensive evaluation of this aspect. This deficiency acts as a constraint on the enhancement and overall development of comprehensive literacy of students. Moreover, the utilization of multimedia technology in vocational institutions holds the potential to significantly enhance teaching innovation and reform [1]. On one hand, it facilitates the creation of a three-dimensional teaching environment, enabling students to engage in learning through multiple senses. This approach stimulates enthusiasm, widens avenues for information acquisition and transmission, and enhances students’ memory, comprehension, and application of knowledge. On the other hand, it supports the transformation of students’ knowledge into practical abilities, thereby augmenting their professional competence. It is evident that a teaching system grounded in multimedia technology offers a more expansive teaching environment and platform for both teachers and students.

Presently, multimedia technology is a new mode of teaching in vocational education for students’ satisfaction and their innovative capabilities [9–11]. The mode of teaching via multimedia technology combines the advantages of online and traditional teaching and learning. The adoption of this teaching approach will significantly progress higher education [12]. Multimedia technology is currently developed and popularized in vocational education [13]. Additionally, there is a growing focus on simulating the efficacy of e-learning mechanisms, taking into account elements like the utilization of online assessment, students’ perceptions of learning and implementation of various instructional strategies [14–16]. Enhancing multimedia technology requires thorough examination and study on students’ satisfaction as well as assessment of the influencing elements to use multimedia technology, especially in vocational colleges of China [17]. The multimedia technology is shown in the following Fig 1.

**Fig 1:** Multimedia technology.

The significance of vocational education through multimedia technology in China is underscored by the transformative potential of innovative approaches, aligning with the evolving needs of the country’s workforce and industries. Several factors contribute to the growing importance of incorporating multimedia technology in vocational education. Many industries in China are experiencing rapid technological advancements. Integrating multimedia technology in vocational education ensures that students are familiar with the latest tools and practices, enhancing their preparedness for real-world applications [12]. Multimedia technology offers a dynamic and interactive learning experience. Incorporating videos, simulations, virtual reality, and other multimedia elements engages students, making the learning process more enjoyable and effective. In an increasingly interconnected world, multimedia technology facilitates access to global knowledge and best practices. Students can benefit from online resources, virtual collaborations, and real-time information, preparing them for globalized industries [8]. Individuals have diverse learning styles, and multimedia caters to visual, auditory, and kinesthetic learners. By incorporating varied multimedia elements, vocational education can accommodate different learning preferences, leading to increased understanding and retention. Multimedia technology is integral to developing skills relevant to the digital age, including digital literacy, information processing, and problem-solving. These skills are essential for success in contemporary workplaces. Multimedia technology allows for the simulation of real-world scenarios, providing students with hands-on experience in a controlled environment. This type of industry-relevant training ensures that graduates are better prepared for the specific challenges of their chosen fields. Industry 4.0, characterized by the integration of digital technologies in manufacturing and other industries, requires a workforce with digital skills. Incorporating multimedia technology in vocational education aligns with the principles of Industry 4.0 and prepares students for the demands of smart manufacturing and automation. By incorporating multimedia technology into vocational education, China can harness the potential of innovative approaches to cultivate a workforce that is not only skilled but also technologically adept and adaptable. This ensures that vocational education remains a key driver of economic growth and competitiveness in the face of evolving industry landscapes and global challenges.

To study the application of multimedia technology to innovative vocational education and its impact on learning satisfaction in China is crucial for several reasons. First, understanding how multimedia technology influences vocational education can help optimize teaching methods. It allows educators to tailor content and delivery methods to improve learning outcomes and student satisfaction [18]. Secondly, China’s educational landscape is evolving rapidly. Studying the role of multimedia technology helps educational institutions adapt to the changing needs of students, industries, and technological advancements, ensuring relevance and effectiveness [19]. Thirdly, multimedia tools have the potential to enhance engagement and improve information retention. Studying their application in vocational education can provide insights into how to create more interactive and effective learning experiences [20]. Fourthly, vocational education aims to prepare students for careers. Assessing the impact of multimedia technology helps ensure that students are equipped with the necessary skills and knowledge demanded by modern industries, improving their employability and job satisfaction [21]. Fifthly, understanding the effects of multimedia technology encourages innovative teaching practices. It fosters the adoption of new teaching methods, such as flipped classrooms, gamification, and interactive learning, which can positively impact student satisfaction [22]. In essence, studying the application of multimedia technology to innovative vocational education in China is vital for improving teaching methods, enhancing learning experiences, aligning education with industry needs, and ultimately, ensuring that students are better equipped for their future careers [23].

In summary, incorporating multimedia technology into vocational education stands as a crucial technological foundation for innovations and satisfaction of students. Given the practical nature of vocational education, students need effective practice, ensuring the comprehensiveness of the learning process. The adoption of computer multimedia technology catalyzes the transformation of teaching and learning of students. The ongoing reforms in vocational institutions, propelled by computer technology, has advanced the field. Therefore, investigating the application of multimedia technology in vocational institutions holds substantial practical significance. It is hypothesized that adoption of multimedia technology causes to innovate and improves the satisfaction of students’ learning in vocational institutions. There is little focus in earlier literature to quantify the impact of multimedia technology for innovations and students’ satisfaction in vocational institutions of China. So this study explores the fundamental ideas and theories about multimedia technology, students’ satisfaction, and innovative capacity in vocational colleges of China. The exploration regarding use of multimedia technology is carried out on 515 students in Chinese vocational institutions using two different formats: online and offline questionnaires. Then impact of each element was examined using multiple linear regression, one-way ANOVA, descriptive statistical analysis, and Pearson’s correlation analysis. It investigates the variables influencing multimedia technology and students’ satisfaction in vocational education and examines the state of affairs and issues surrounding students’ contentment with it from creative angles. In order to optimize teaching quality and advance multimedia technology reform, it is crucial that the study delves further into the direction and focus of multimedia technology improvement.

## 2. Theoretical framework

The theoretical framework of this research provides the conceptual foundations. The study is drawn from the constructivist learning theory, which posits that learning is an active process where individuals construct knowledge based on their experiences. In the context of vocational education, this theory suggests that incorporating multimedia technology can facilitate hands-on, interactive learning experiences, allowing students to construct their understanding of the subject matter. The Technology Acceptance Model (TAM) is also integrated to understand how students’ perceptions of multimedia technology influence their acceptance and usage. This model suggests that perceived ease of use and perceived usefulness of technology impact user attitudes and, consequently, their behavioral intentions. In this case, it could be applied to assess students’ attitudes towards and satisfaction with the use of multimedia technology in vocational education. Cognitive Load Theory is also relevant to assess the mental effort required for learning tasks. Multimedia technology, if not appropriately designed, could impose excessive cognitive load, hindering learning satisfaction. The theory helps in understanding how the cognitive load imposed by multimedia elements affects learning outcomes and satisfaction. The Experiential Learning Cycle, as proposed by David Kolb, emphasizes the importance of concrete experience, reflective observation, abstract conceptualization, and active experimentation in the learning process. Multimedia technology can be seen as a tool that facilitates each stage of this cycle, enhancing the overall learning experience and potentially contributing to higher satisfaction. Social Cognitive Theory, developed by Albert Bandura, emphasizes the role of observational learning, imitation, and modeling in the learning process. In the context of vocational education, multimedia technology can provide opportunities for students to observe and learn from realistic scenarios, contributing to their satisfaction with the learning process. The theoretical model is shown in the following Fig 2.

**Fig 2:** Theoretical model.

Motivation theories, such as Self-Determination Theory, may be applied to understand how multimedia technology influences students’ intrinsic motivation and satisfaction. The theory posits that autonomy, competence, and relatedness are essential for motivation. Multimedia technology, if designed to support these psychological needs, could enhance students’ satisfaction and engagement. Innovation Diffusion Theory can be incorporated to understand how the adoption and diffusion of multimedia technology occur within the context of vocational education. This theory explores the stages of innovation adoption, from awareness to adoption, and can help identify factors influencing the successful integration of multimedia technology. Human-Computer Interaction principles guide the design and evaluation of multimedia technology in vocational education. These principles focus on creating user-friendly and effective interactions between humans and computers, contributing to overall satisfaction with the technology. By integrating these theoretical perspectives, the research can develop a robust framework that not only guides the study but also contributes to a deeper understanding of the complex relationships between multimedia technology, innovative vocational education, and learning satisfaction in the Chinese context.

In recent years, the widespread adoption of information technology in colleges and universities has led to the incorporation of hardware facilities. Teachers continuously enhance their skills, ensuring that educational institutions possess both hardware and software resources capable of offering adequate support for multimedia and network technology. Multimedia technology meets the presentation demands of vocational education. The audiovisual features of multimedia courseware effectively engage students’ enthusiasm and sensory perception. Through the integration of multimedia and network technology, vocational education teaching encompasses both theoretical and practical components. Leveraging multimedia and internet technology provides a wealth of images, pictures, and information, enhancing the breadth of content in vocational education and fostering its integration into society.

On the basis of above discussion, following hypotheses are developed.

H 1: The use of multimedia technology significantly affects the innovative capability of students in vocational institutions.
H 2: Adoption of multimedia technology positively affects the students’ learning in vocational institutions.

## 3. Literature review

### 3.1 Multimedia technology

Research on multimedia technology in China encompasses a wide range of studies exploring its application and impact across various educational contexts [24]. Researchers investigate how multimedia technology affects learning outcomes in different educational settings. This includes assessing its influence on knowledge retention, comprehension, and academic achievement among students in vocational, higher education, and K-12 settings [25]. Studies delve into innovative pedagogical approaches involving multimedia technology. They explore how educators incorporate multimedia tools into teaching methods, such as flipped classrooms, blended learning models, gamification, and interactive learning environments [26]. Research focuses on the integration of multimedia technology into vocational education programs [27]. This involves examining its role in practical skill development, industry alignment, and preparing students for specific job requirements in diverse vocational fields [12, 18]. Researchers analyze the relationship between multimedia technology and student satisfaction [28]. They explore how the use of multimedia tools impacts student engagement, motivation, and overall satisfaction with the learning process in Chinese educational settings. Studies investigate adaptive learning systems utilizing multimedia technology [15, 29]. They explore how these systems cater to individual learning styles, adapt content delivery, and provide personalized learning experiences for students in China. Research focuses on the accessibility of multimedia technology in education, particularly for students with diverse needs and in remote areas of China. Studies examine how to make multimedia resources more accessible and inclusive for all learners [22, 30]. Researchers explore how multimedia technology fosters innovation and creativity among students [31]. They investigate how creative projects, content creation tools, and collaborative multimedia platforms enhance students’ creative thinking and problem-solving skills [19]. Some studies concentrate on training educators in the effective use of multimedia technology [20, 32]. They assess the impact of professional development programs on educators’ ability to integrate multimedia tools into their teaching practices [16, 33]. Research in this area focuses on policy frameworks and strategies for successful implementation of multimedia technology in Chinese educational institutions [34]. This includes analyzing policies, guidelines, and best practices to optimize technology integration. Studies evaluate specific multimedia tools, platforms, or applications used in Chinese educational contexts [19, 25]. This involves assessing the effectiveness, usability, and impact of these tools on teaching and learning outcomes [11]. Overall, research on multimedia technology in China’s educational landscape spans various dimensions, aiming to understand its effectiveness, optimize its implementation, and enhance the overall quality of education across different levels and disciplines.

### 3.2 Students’ learning satisfaction

At the end of the 20th century, academicians formally brought the idea of student satisfaction in the area of education—which is based on consumer satisfaction. Higher education has paid more attention to meeting students’ expectations and needs as a result of growing awareness about requirements and expectations which are similar to those of services industry [35]. A key factor in assessing the quality of instruction is the students’ learning experience and contentment, who are the subjects of education [29]. Diverse scholarly perspectives have led to differing interpretations of what constitutes learning satisfaction [13]. One is the concept of disparity derived from comparing the pre- and post-learning of students. It is the degree to which students’ psychological satisfaction—or lack thereof—with the quality of instruction during the teaching process is compared to their pre-learning demands or expectations. The concept of student satisfaction [36] emphasizes satisfaction at various levels, such as those related to living arrangements, physical facilities, educational strategies, and so forth. It also includes other components as an extension and enhancement of the holistic concept, including perception of connection, and support for learning [21].

A substantial amount of research indicates that students are more satisfied with multimedia technology than they are with traditional learning environments [37–40]. According to research on the variables that affect the satisfaction of students with multimedia technology, having constant access to the instructor is thought to be crucial [32, 36]. Some students claim that compared to traditional courses, they receive instructor feedback and their grades more quickly [26, 32]. The study [29] looked into the attitudes, relationships, and interactions of 140 TEFL students with the quality of blended learning. They discovered that students had the biggest impact coefficient on teaching quality and satisfaction and were most satisfied with teacher-student interaction in blended learning. Among them, the teaching aptitude of the teachers greatly outweighed the attitude of the teachers in terms of satisfaction [32]. It is also found that the main factors influencing students’ learning satisfaction are “self-efficacy, performance expectations, system functions, content characteristics, interaction, and learning atmosphere” [41]. Teacher-student contact also has a significant impact on learning atmosphere.

### 3.3 Research on constructivist learning theory

Piaget, a Swiss educationalist, developed a theory of children’s cognitive development. Piaget’s individual constructivism and Vygotsky’s social constructivism are now widely recognized as components of constructivist learning theory [42]. Constructivism has become a potent paradigm for illuminating how people pick up new knowledge and learn about the world around them [16, 31, 39]. In line with this theory, learners construct their own cognitive, meaning that the formation of their own knowledge and the development of cognitive structures are essentially personal and dependent on the learner’s interaction with the surrounding environment rather than the educator’s face-to-face instruction [43]. Building cognitive frameworks emphasizes the subjectivity of the learner by the learner actively absorb knowledge rather than passively [44]. According to constructivist learning theory, learners constantly create and modify their own knowledge systems, and the learning environment is vital to this process [23, 36]. The learning environment, which consists of four main components—"scenario," "cooperation," "conversation," and "meaning construction"—influences people who wish to better design a learning system that aligns with their own [45]. In multimedia technology, students change from being passive recipients of knowledge from their teachers to active constructors through the ongoing interaction of their prior knowledge with newly acquired information, replacing the teacher’s one-sided knowledge transmission that occurs in traditional instruction [29]. Multimedia technology stimulates students’ curiosity about learning, makes them take an active role in their education, and fosters their participation and initiative in communication and interaction [27, 46].

Constructivist theory has implications for instructional design, curriculum development, and assessment practices, emphasizing the creation of learning environments that encourage exploration, collaboration, and the active construction of knowledge [47]. It aligns with a student-centered approach to education, emphasizing the importance of fostering a learner’s intrinsic motivation and curiosity. Constructivism posits that learning is a process of mental construction where individuals build upon their prior knowledge and experiences to make sense of the world. It suggests that learners actively create their own understanding by engaging with new information, connecting it to what they already know, and refining their mental models through experience and reflection [47, 48]. Key principles of constructivism include active engagement, the importance of prior knowledge, social interaction, scaffolding, the Zone of Proximal Development (ZPD), discovery learning, reflection, authentic tasks, consideration of multiple perspectives, and individualized learning paths. Constructivism has had a significant impact on educational philosophy and instructional practices, influencing the design of learner-centered environments that encourage critical thinking, collaboration, and the application of knowledge in real-world contexts.

Constructivism originates from instructional methods, aiming to explore how various interactive exercises prompt independent learning of students and defining the role of teachers in learning process. The primary goal of constructivist teaching is to cultivate students who possess enduring learning capabilities, emphasizing a shift in perspective from the teacher to the student. This approach underscores the dynamic generation of new knowledge through the restructuring of existing information, challenging traditional educational paradigms. This paper delves into the ways in which constructivism shapes learning in vocation institutions by considering the role of multimedia technology. Constructivism encourages students to form new understandings by integrating existing knowledge [49]. Rooted in an epistemology that appreciates diverse ways of thinking [44], constructivism emphasizes the learner’s agency and views learning as a social, interactive process. The central concept of constructivist theory is that, despite disruptions caused by conflicts or unexpected developments, the cognitive entity strives to develop and maintain equilibrium [50]. Three fundamental types of constructivism are recognized: cognitive constructivism based on Piaget, social constructivism based on Vygotsky, and radical constructivism. Cognitive constructivism emphasizes on the role of cognitive processes in learning and understanding how individuals actively construct knowledge through mental activities. In this type of constructivism, learning is viewed as a personal, internal process where individuals actively construct their own understanding [51]. This process involves mental activities such as problem-solving, critical thinking, and reflection. Cognitive development outlines distinct stages through which individuals progress. These stages, including the sensorimotor, preoperational, concrete operational, and formal operational stages, represent different levels of cognitive abilities and understanding. Cognitive constructivism also supports the idea of discovery learning, where learners actively explore and experiment to discover concepts on their own. This hands-on, experiential approach is believed to enhance understanding and retention. While closely associated with social constructivism, the idea of scaffolding, where more knowledgeable individuals provide guidance and support to learners, is also present in cognitive constructivism. However, the emphasis is on the individual’s internal cognitive processes [52].

Social constructivism emphasizes on the social and collaborative aspects of knowledge construction. It builds upon the broader constructivist framework, incorporating the idea that learning is not only an individual cognitive process but is also shaped by social interactions and cultural contexts. Interactions with others, such as peers, teachers, and more knowledgeable individuals, play a crucial role in shaping an individual’s understanding of the world [53]. The concept of the Zone of Proximal Development is introduced, which represents the gap between what a learner can do independently and what they can achieve with guidance or assistance. Social interactions within the ZPD facilitate learning and development. Collaborative learning is a fundamental aspect of social constructivism. Learners work together to solve problems, discuss ideas, and construct knowledge collectively. Collaboration fosters diverse perspectives and shared understanding [54].

Radical constructivism is a philosophical and educational perspective that extends the principles of constructivism to emphasize the subjective and individual nature of knowledge construction. It is often associated with the work of Ernst von Glasersfeld [48]. Unlike other forms of constructivism, radical constructivism places a strong emphasis on the idea that knowledge is actively created by individuals based on their unique experiences and interactions with the environment. There is an emphasis on understanding the world from the learner’s point of view. Learners are considered autonomous agents who actively interpret and organize their experiences. Reality is seen as a mental construct rather than an objective external reality [55]. According to radical constructivism, individuals do not have direct access to an objective reality; rather, they interpret and create their understanding of the world. Learning is viewed as a continuous process of adaptation and accommodation. Individuals continually adjust their mental models to make sense of new experiences and information, leading to ongoing cognitive development. Radical constructivism acknowledges the importance of interactions with the environment in shaping individual understanding [56]. However, it places greater emphasis on the individual’s interpretation of those interactions rather than on the objective properties of the external world. In conclusion, the adaptive learning system suggests that a collection of conceptually distinct systems can be created by efficiently classifying learning components. In light of the study’s focus and issue, the pertinent influencing elements are analyzed and arranged into four categories in this study: learning, teaching, curriculum, and innovative capacity [18, 25, 47]. Learning behaviors and attitudes are included in the learning component. Teaching abilities, teaching strategies, and teaching attitudes are all included in the teaching dimension. Platform and curriculum design are included in the curriculum dimension [48]. The innovative capacity covers the dimensions of skill acquisition, knowledge retention, and collaboration and communication [21]. The findings of this research may be used for better decision making when implementing multimedia technology, and effectively achieving more meaningful learning in vocational colleges of China.

## 4. Materials and methods

The approval from research ethics committee of Beijing Institute of Management and Economics is gained prior to conducting the study vide no. BIEM/REC/2023/205. A written consent was gained from participants of the study to participate and publish this study. In order to guarantee the accuracy of the data sample, a questionnaire survey was carried out through online sources between July 2023 and October 2023 among vocational college students with multimedia technology learning experiences in China. Out of the 680 questionnaires that were delivered, 515 were deemed appropriate for empirical analysis. The descriptive statistics are given in Table 1.

**Table 1:** Demographic analysis (N = 515).

Item	Sub-Item	Frequency	Percentage
Gender	Male	265	51.46
	Female	250	48.54
Educational Level	Freshman	198	38.45
	Sophomores	158	30.68
	Juniors	86	16.70
	Seniors	73	14.17
Marital Status	Unmarried	388	75.34
	Married	127	24.66
Age	18–20 years	201	39.03
	21–23	198	38.45
	24 and More	116	22.52

### 4.1. Questionnaire design

The targeted and quantitative design of the questionnaire was achieved by referencing pertinent studies and incorporating them with the real state of multimedia technology in Chinese vocational institutions [12, 23, 28, 35, 46]. The study’s scale design is broken down into two phases: first, ongoing adjustments are made after consulting with experts and instructors who use multimedia technology in vocational colleges and incorporating the suggestions and opinions of students who have used the technology; In order to make sure that each indicator’s significance level was less than 0.05, a pre-survey was carried out to distribute questionnaires. Respondents were allowed to select the option that best suited their real-world circumstances from a five-point Likert scale, where scores range from one to five.

### 4.2. Exploratory factor analysis and validity testing

The optimal impact of factor analysis occurs when KMO (Kaiser-Meyer-Olkin) > 0.9. The exploratory factor analysis results are good, as evidenced by the test results of various question items, which show that the total KMO value of the questionnaire is 0.981 > 0.9, the Sig value is 0.01 < 0.05, the cumulative explained variance is 78.83%, and the variance explained after rotation of each factor was above 10%. Each factor’s factor loading coefficient is greater than 0.6, which show strong scale validity. Table 2 presents the empirical results.

**Table 2:** Validity of questionnaire.

Cumulative Explained Variance		78.83
KMO		0.981
Bartlett’s test	Chi-square	22153.24
	df	225
	Sig.	0.01

Cronbach’s alpha reliability analysis is used in this work. The three dimensions—students, teachers, and curriculum—have Cronbach’s alpha values of 0.926, 0.932, and 0.958, respectively; the fourth part’s Cronbach’s alpha value is 0.963, reflecting the fact that all dimensions have alpha coefficients that are greater than 0.9, indicating that the questionnaire has strong reliability.

## 5. Estimated results

According to survey data, the average satisfaction level with multimedia technology is in the upper-middle level, at 4.38. Three of these metrics were agreed upon or strongly agreed upon by over 72% of the students, indicating a high level of satisfaction with multimedia technology in vocational colleges. More than half of the students are satisfied with the learning objectives. The students who agree and strongly agree with the indicator "In general, I am satisfied with the multimedia technology" are the most, reaching 73.9%, and the students who agree and strongly agree with the indicator "By studying this course, I have completed the expected learning objectives or tasks" are 61.3%.

College students are the least content with their own learning status, according to the results of the satisfaction survey for the three areas of teaching, learning, and curriculum. Their satisfaction with their own attitudes and behaviors clearly varies, which reflects the discrepancy between knowing and acting. It is clear that teachers’ methods and abilities need to be further optimized because students’ contentment with teachers’ teaching attitudes is higher on average than their satisfaction with methods and abilities. The hours and frequency of instruction, the design of the teaching materials, and the curriculum all fall short of adequately meeting the needs of the students.

Table 3 displays the findings of the one-way ANOVA and independent sample t-test analyses of the satisfaction variability based on the individual characteristics of vocational college students. The results indicate that there is no significant difference between the satisfaction of the various personality characteristics, with a significant p-value of larger than 0.05.

**Table 3:** Differential analysis.

Characteristics	Category	Mean Value	SD	F-value
Gender	Male	3.49	0.91	1.83
	Female	3.85	0.85	
Educational Level	Freshman	3.63	0.92	1.76
	Sophomores	4.01	0.87	
	Juniors	3.89	0.85	
	Seniors	3.85	0.83	
Marital Status	Unmarried	4.02	0.81	1.82
	Married	3.69	0.76	
Age	18–20 years	3.87	0.83	1.74
	21–23	3.85	0.74	
	24 and More	3.96	0.85	
**Students’ Satisfaction with Multimedia Technology and Learning Platforms**				
Super star learning	Not Selected	3.69	0.85	1.82
	Selected	3.52	0.84	
MOOC	Not Selected	3.64	0.79	1.76
	Selected	3.43	0.83	
Ding Talk	Not Selected	3.67	0.81	1.86
	Selected	3.51	0.87	
Other	Not Selected	3.09	0.88	1.92
	Selected	4.02	0.82	
**Multimedia Technology and Innovative Vocational Education**				
Skill Acquisition	Not Selected	4.01	0.79	1.87
	Selected	4.21	0.81	
Retention of Information	Not Selected	3.89	0.83	1.75
	Selected	3.76	0.74	
Collaboration and Communication	Not Selected	3.67	0.88	1.84
	Selected	4.03	0.83	
**Multimedia Technology With Different Teaching Methods**				
Teacher-Led Lectures	Not Selected	3.85	0.82	7.69***
	Selected	3.76	0.79	
Mutual Discussions	Not Selected	3.59	0.84	9.58***
	Selected	3.75	0.82	
Student-Led Lectures	Not Selected	3.82	0.83	9.83***
	Selected	3.69	0.76	

Table 3 displays the results of a one-way ANOVA on student satisfaction with instruction across various learning platforms and the function of multimedia technology in creative vocational education. The findings indicate that, regardless of the learning platform, there is no discernible variation in students’ satisfaction with multimedia technology. However, because of various online resources, there is a notable variation in students’ satisfaction with multimedia technology. Students prefer online learning environments with teacher-built, organized courses over those with fragmented courseware. Enhancing face-to-face instruction with technology has the potential to increase student engagement and boost academic performance. Multimedia technology at vocational institutions generally deals more with augmentation, modification, and substitution than with redefinition. Significant variations were discovered in the comparison analysis of the students’ satisfaction levels with multimedia technology. Students preferred peer-to-peer discussions and lectures led by students. These two instructional approaches have strengthened their relationship, increased student involvement, interaction, and communication, given students greater initiative, and made it simpler for teachers to keep an eye on their progress and status. Student satisfaction with multimedia technology varied significantly depending on the type of online instruction used.

Pearson correlation analysis and multiple linear regression are applied. The goal was to investigate the relationship between student satisfaction and factors of the learning dimension, teaching dimension, innovative capacity, and curriculum dimension of multimedia technology in vocational colleges. Table 4 displays the findings of correlation analysis.

**Table 4:** Correlation matrix.

	Students’ Satisfaction	Learning Dimension	Teaching Dimension	Curriculum Dimension	Innovative Capacity
Students’ Satisfaction	1				
Learning	0.47**	1			
Teaching	0.42**	0.48**	1		
Curriculum	0.51**	0.43**	0.39**	1	
Innovative Capacity	0.52**	0.47**	0.46**	0.39**	1

All dimensions are significantly positively correlated with students’ satisfaction with multimedia technology, according to the results of the correlation analysis. This means that an increase in student satisfaction with themselves, teachers, and curriculum will be followed by an increase in satisfaction with multimedia technology and an increase in innovative capacity. The p-values corresponding to the satisfaction of multimedia technology and all other factors are all close to 0. Since the correlation coefficients are below 0.70, the phenomena of multicollinearity does not exist.

### 5.1. Regression analysis

There are noteworthy correlations between the variables according to the correlation analysis. The study’s independent variables, such as the learning dimension (learning attitude, learning behavior), the teaching dimension (teaching attitude, teaching method, teaching ability), and the curriculum dimension (course design, platform design), can all reflect changes in teachers’ satisfaction with their work, as demonstrated by the results in Table 5. There is a substantial linear association between the independent factors and the dependent variable, which is satisfaction with multimedia technology, according to the regression model’s F-value and significance level. The elements that have the biggest effects on students’ satisfaction with multimedia technology are, thus, learning attitudes, course design, teaching strategies, and innovative ability.

**Table 5:** Regression analysis.

	Satisfaction with Multimedia Technology
**Learning Dimension**	
Learning Attitude	0.23***
Learning Behavior	0.21**
**Teaching Dimension**	
Teaching Attitude	0.16***
Teaching Method	0.17***
Teaching Ability	0.19***
**Curriculum Dimension**	
Course Design	0.22***
Platform Design	0.19***
**Innovative Capacity**	
Skill Acquisition	0.25***
Retention of Information	0.26***
Collaboration and Communication	0.19***
B	2.36
F	125.21***
Adjusted R^2^	0.65

## 6. Discussion

This study investigates the relationship among multimedia technology, students; learning and their innovative vocational education in China. The findings of the study reveal that the relationship between multimedia technology and student learning is inherently positive, offering numerous benefits that enhance the learning experience in various ways. Multimedia technology makes learning more interactive and engaging [49]. Visuals, videos, simulations, and interactive elements capture students’ attention and interest, keeping them more engaged in the learning process compared to traditional methods [16, 50]. This engagement leads to better focus and improved retention of information. Students have diverse learning styles, and multimedia technology accommodates these differences [34, 51]. Visual learners benefit from graphics and videos, auditory learners from audio recordings or lectures, while kinesthetic learners benefit from interactive simulations and hands-on activities. This variety ensures that the needs of different learners are met. Multimedia aids in better understanding and retention of information [29, 52]. Concepts that are complex or abstract can be explained more effectively through multimedia tools, as they offer visual representations and real-life examples, making learning more tangible and easier to grasp [53]. Multimedia technology allows students to learn at their own pace. They can pause, rewind, or review materials as needed, ensuring a deeper understanding of the content before moving forward [54]. This autonomy fosters a more personalized learning experience. Multimedia tools facilitate practical application of knowledge [30, 55]. Simulations and virtual labs provide opportunities for students to apply theoretical concepts in simulated real-world scenarios, enhancing their understanding through practical experience [56]. Interactive and visually stimulating content tends to increase students’ motivation to learn. Multimedia technology can make learning more enjoyable and interesting, motivating students to explore topics further and take a more active role in their education [32, 44]. Multimedia tools promote collaboration among students and facilitate communication with instructors [28]. Online forums, virtual classrooms, and collaborative projects enable students to engage in discussions, share ideas, and work together, fostering a sense of community and enhancing learning through peer interaction [57]. Multimedia technology offers flexibility in accessing learning materials. Students can access resources anytime, anywhere, allowing for learning beyond traditional classroom hours [31, 58]. This flexibility accommodates different schedules and learning preferences, making education more accessible. Multimedia tools enable immediate feedback on students’ progress. Assessments, quizzes, and interactive exercises can provide instant feedback, allowing students to identify areas for improvement and take corrective actions promptly [24, 59]. In a world reliant on technology, exposure to multimedia tools equips students with digital literacy skills essential for their future careers. Familiarity with multimedia technology enhances their adaptability in an increasingly tech-driven workforce [35, 60]. In summary, multimedia technology enriches the learning process by increasing engagement, accommodating diverse learning styles, improving comprehension, enabling self-paced learning, fostering practical application, boosting motivation, facilitating collaboration, providing flexibility, offering instant feedback, and preparing students for the digital era [31, 46]. This positive relationship between multimedia technology and student learning is instrumental in creating a more effective and enriching educational experience.

Multimedia technology has significantly impacted innovative vocational education by revolutionizing the way information is delivered, skills are acquired, and learning experiences are enhanced [16, 61]. Multimedia tools offer an interactive and engaging learning environment. They provide dynamic content, such as videos, simulations, and interactive modules, which captivate students’ attention and cater to diverse learning styles [39, 62]. This engagement fosters better focus, leading to improved information retention and understanding. Multimedia technology enables on-demand access to educational resources, breaking geographical barriers and time constraints [26, 63]. Students can learn at their own pace, revisit materials, and access a variety of learning materials, accommodating different learning speeds and preferences. It offers a multi-sensory experience, combining visuals, audio, and interactive elements to create a richer learning experience [64]. For vocational education, this means the ability to simulate real-world scenarios, provide virtual hands-on experiences, and offer practical, industry-relevant training in a controlled environment [55]. Multimedia tools facilitate hands-on learning experiences [44]. Through simulations, virtual labs, and interactive tutorials, students can practice skills in a risk-free environment. For vocational training, this is especially beneficial as it allows for the development of practical skills necessary for various professions [65]. These technologies allow for personalized learning pathways, catering to individual student needs. Adaptive learning systems can assess strengths and weaknesses, offering customized content and pacing to optimize learning outcomes. Multimedia technology fosters collaboration among students and instructors [36]. Features like discussion forums, virtual classrooms, and collaborative projects enable interaction, peer learning, and real-time feedback, creating a collaborative learning community. It stimulates creativity by offering tools for content creation and expression [66]. Students can produce multimedia projects, presentations, and portfolios that showcase their skills and creativity, encouraging innovative thinking and problem-solving abilities. Vocational education benefits greatly from multimedia technology’s ability to replicate real-world scenarios [39]. This technology allows students to gain practical experience and exposure to industry-specific tools and environments, better preparing them for their future careers. Multimedia tools offer opportunities for continuous assessment and feedback [58]. Educators can track progress, assess performance, and adapt teaching strategies based on real-time data, ensuring continuous improvement in the learning process [67–70]. While initial setup costs may exist, multimedia technology often proves cost-effective in the long run. Digital resources can be reused, updated, and distributed at a lower cost compared to traditional learning materials, making education more sustainable and accessible [31]. Multimedia technology has fundamentally transformed vocational education by making it more engaging, accessible, practical, and tailored to individual needs [28]. Its integration has not only enhanced the learning experience but also aligned education more closely with industry requirements, better preparing students for the workforce [68, 71–74].

Multimedia technology offers several avenues through which it enhances the satisfaction of Chinese students in vocational colleges. Multimedia tools create an interactive and immersive learning atmosphere. In vocational colleges, where practical skills are emphasized, these tools can simulate real-world scenarios, making the learning experience more engaging and applicable [61]. Multimedia technology provides access to a wide array of resources like videos, interactive modules, virtual labs, and online lectures [69, 75]. This variety caters to diverse learning styles and preferences, allowing students to explore content in ways that suit them best. Customization is a key benefit of multimedia tools [55]. Chinese students in vocational colleges can access tailored content that matches their learning pace, interests, and skill levels, contributing to a more satisfying and effective learning journey. Visual and interactive elements in multimedia aid in better understanding and retention of complex concepts. This is particularly beneficial in vocational colleges where technical knowledge is vital and multimedia technology helps in clarifying intricate subjects. Practical skills are fundamental in vocational education [41]. Multimedia technology offers opportunities for hands-on learning through simulations, virtual labs, and interactive tutorials, allowing students to practice and refine skills in a controlled environment [23, 76]. Multimedia tools facilitate collaboration among students and instructors. Chinese students can engage in group projects, online discussions, and virtual classrooms, fostering effective communication, knowledge sharing, and peer learning [70, 77]. Vocational colleges aim to prepare students for specific industries [39]. Multimedia technology bridges the gap between academia and industry by exposing students to relevant tools, technologies, and practices, making them more job-ready and satisfied with their education. Multimedia technology encourages innovative thinking and creativity among students [17, 78, 79]. By providing tools for content creation and expression, students can showcase their skills in projects, presentations, and portfolios, enhancing their satisfaction with the learning process [36, 80]. In conclusion, the integration of multimedia technology in vocational colleges for Chinese students greatly enhances satisfaction by creating an engaging, personalized, practical, and industry-aligned learning experience that equips them with relevant skills for their chosen careers.

### 6.1 Implications

The implications derived from the study span various realms, each offering insights for stakeholders and policymakers. The findings underscore the need for strategic policy reforms that promote the integration of multimedia technology within vocational education curricula. Policymakers should consider allocating resources and formulating guidelines to encourage the widespread adoption of multimedia tools in vocational institutions. Institutions should invest in robust technological infrastructure to ensure equitable access to multimedia resources across diverse geographical and socio-economic regions in China. Bridging the digital divide is crucial for providing equal learning opportunities to all vocational students. There is a clear need for comprehensive training programs aimed at equipping educators with the necessary skills to effectively utilize multimedia technology in their teaching methods. Continuous professional development initiatives can empower educators to maximize the benefits of multimedia tools. The study highlights the importance of fostering stronger ties between vocational institutions and industries. Collaborative efforts can ensure that curriculum content aligns with industry needs, enhancing students’ preparedness for the workforce. Institutions should explore methods to further customize learning experiences through multimedia technology. Tailoring content to match individual learning styles and preferences can significantly enhance learning satisfaction and outcomes. Emphasis should be placed on leveraging multimedia tools to enhance practical skill development. This involves providing more hands-on experiences and simulations that mimic real-world vocational scenarios. Encouraging innovation in the use of multimedia technology is vital. Institutions should create an environment that fosters experimentation and creative application of these tools to continually enhance vocational education. Overall, the implications derived from the study emphasize the need for comprehensive strategies that harness the potential of multimedia technology to transform vocational education in China, ensuring higher levels of learning satisfaction and better preparedness for the evolving job market.

The study points towards avenues for further research, including longitudinal studies to assess the long-term impact of multimedia technology on vocational students’ career success and exploring emerging technologies for even more effective integration into vocational education.

## 7. Conclusion

This study highlights the multifaceted impact of integrating multimedia technology into vocational education and its influence on learning satisfaction among vocational students of China. The novelty and uniqueness of the study lie in its specific focus on multimedia technology in the context of vocational education in China, its emphasis on innovation, the assessment of learning satisfaction, consideration of the Chinese educational landscape, and its potential contributions to both the educational technology literature and policy discussions. This study contributes to literature by focusing specifically on the application of multimedia technology in the context of vocational education in China. This specificity acknowledges the unique challenges, opportunities, and characteristics of vocational education within the Chinese educational system, making the study contextually relevant. This study also explores the innovative integration of multimedia technology into vocational education. This approach recognizes the potential of multimedia tools to transform traditional teaching methods and enhance the learning experience in vocational settings. The emphasis on innovation highlights a departure from conventional practices. Investigating how multimedia technology influences students’ satisfaction with their learning experiences provides valuable insights into the effectiveness of this innovative approach. Learning satisfaction is a crucial factor in understanding the overall success of educational interventions. This consideration adds depth and specificity to the research. The study contributes to the broader field of educational technology literature by examining the application of multimedia technology in a vocational education context. By focusing on China, it may offer insights and recommendations that are valuable not only for practitioners in China but also for educators and researchers globally seeking to enhance vocational education through technology.

Through comprehensive analysis and empirical exploration, some key conclusions are drawn. The incorporation of multimedia technology has significantly enriched the learning experience in vocational education across various disciplines in China. The availability of interactive tools, simulations, and virtual labs has created a dynamic and engaging educational environment. There is a clear positive correlation between the use of multimedia technology and heightened levels of learning satisfaction among vocational students in China. The diverse and interactive nature of multimedia tools has positively impacted students’ engagement, motivation, and overall enjoyment of the learning process. Multimedia technology has effectively facilitated practical skill development, providing students with hands-on experiences that simulate real-world scenarios. This hands-on approach has contributed to higher levels of competence and confidence among students in vocational fields. The integration of multimedia technology in vocational education programs has successfully aligned curriculum content with the evolving needs of industries in China. Students are better prepared for the demands and requirements of their respective vocational fields, enhancing their employability and career readiness. The customization offered by multimedia tools has allowed for tailored learning experiences, accommodating diverse learning styles and preferences. This flexibility has empowered students to pace their learning according to individual needs, contributing to higher levels of satisfaction and understanding. While the benefits of multimedia technology in vocational education are evident, challenges such as access disparities, training needs for educators, and the constant evolution of technology must be addressed. Leveraging these challenges as opportunities for further enhancement is critical for sustained growth. In conclusion, the study underscores the pivotal role of multimedia technology in shaping innovative vocational education in China. Its positive impact on learning satisfaction, practical skill development, industry alignment, and customized learning experiences underscores the significance of continued investment and strategic integration of multimedia tools within vocational educational frameworks. Embracing this integration can further elevate the quality of vocational education, ensuring that students are equipped with the skills and satisfaction necessary for success in their future careers.

## Supporting information

S1 Data (XLSX)
